# Artificial Intelligence Smartphone Application for Detection of Simulated Skin Changes: An In Vivo Pilot Study

**DOI:** 10.1111/srt.70056

**Published:** 2024-10-04

**Authors:** Gabriela Lladó Grove, Gorm Reedtz, Brian Vangsgaard, Hassan Eskandarani, Merete Haedersdal, Flemming Andersen, Peter Bjerring

**Affiliations:** ^1^ Department of Dermatology Copenhagen University Hospital – Bispebjerg Copenhagen Denmark; ^2^ Department of Dermatology Private Hospital Molholm Vejle Denmark; ^3^ Department of Dermatology Aalborg University Hospital Aalborg Denmark; ^4^ SkinChange.AI Aps Vejle Denmark; ^5^ Department of Clinical Medicine University of Copenhagen Copenhagen Denmark

**Keywords:** AI, artificial intelligence, detection, feasibility study, pilot study, skin change, smartphone

## Abstract

**Background:**

The development of artificial intelligence (AI) is rapidly expanding, showing promise in the dermatological field. Skin checks are a resource‐heavy challenge that could potentially benefit from AI‐tool assistance, particularly if provided in widely available AI solutions. A novel smartphone application(app)‐based AI system, “SCAI,” was developed and trained to recognize spots in paired images of skin, pursuing identification of new skin lesions. This pilot study aimed to investigate the feasibility of the SCAI‐app to identify simulated skin changes in vivo.

**Materials and methods:**

The study was conducted in a controlled setting with healthy volunteers and standardized, simulated skin changes (test spots), consisting of customized 3‐mm adhesive spots in three colors (black, brown, and red). Each volunteer had a total of eight test spots adhered to four areas on back and legs. The SCAI‐app collected smartphone‐ and template‐guided standardized images before and after test spot application, using its backend AI algorithms to identify changes between the paired images.

**Results:**

Twenty‐four volunteers were included, amounting to a total of 192 test spots. Overall, the detection algorithms identified test spots with a sensitivity of 92.0% (CI: 88.1–95.9) and a specificity of 95.5% (CI: 95.0–96.0). The SCAI‐app's positive predictive value was 38.0% (CI: 31.0–44.9), while the negative predictive value was 99.7% (CI: 99.0–100).

**Conclusion:**

This pilot study showed that SCAI‐app could detect simulated skin changes in a controlled in vivo setting. The app's feasibility in a clinical setting with real‐life skin lesions remains to be investigated, where the challenge with false positives in particular needs to be addressed.

**Abbreviations**
3D: three‐dimensional
AI: artificial intelligence
app: application
CI: confidence intervals
CNN: convolutional neural network
iOS: iPhone Operation System
ISO: International Organization for Standardization
LED: light emitting diode
NPV: negative predictive value
PPV: positive predictive value
SCAI: SkinChange.AI, a smartphone application‐based AI system

## 1 Introduction

Amid the rapidly growing field of artificial intelligence (AI) in the medical sector, there is a potential for new applications in dermatology, ranging from skin conditions such as acne and eczema to skin aging and skin cancer [1, 2, 3, 4, 5]. Skin changes and appearance of new skin lesions is a common concern, and while keeping track may be crucial, it is also a time‐dependent and resource‐heavy endeavor [6, 7]. It is asserted that AI tools may contribute to making detection of skin changes increasingly accessible, especially where resources are sparse [8, 9].

The field of smartphone applications for skin checks is exploding and there is a consumer‐driven interest in providing new solutions [10]. However, the requirements for such tools are substantial and include handiness, widespread availability, and low cost, as well as being scientifically well‐founded with studies backing their applicability [11, 12].

Upcoming AI‐system developments mainly circle around lesion‐specific features based on clinical or dermoscopic images [7, 13–17]. In contrast, there are fewer solutions providing AI tools for nondiscriminatory identification of skin changes over time [18, 19]. Such tools could be helpful for general skin checks, particularly of large or unattainable skin areas, and in skin types with multiple skin lesions.

A novel smartphone application (app)‐based visual AI system, SkinChange.AI (SCAI), has been developed in the pursuit of AI‐assisted identification of skin changes over time. The SCAI‐app has been trained with open‐source AI to non‐discriminatorily identify spots on skin. This is in contrast to many available AI tools that rely on a large photo library with validated skin lesions, histology, imaging, or dermoscopy [20, 21]. In addition, a common challenge in application of AI tools is the quality of images, as the collection of standardized images can be very operator‐dependent. In anticipation of this, the SCAI‐app provides both app‐based and AI‐assisted standardization of paired images of skin. However, the SCAI‐app's feasibility in terms of sensitivity and specificity to detect new spots on skin remains to be tested. This pilot study aimed to investigate the feasibility of the SCAI‐app for identification of simulated skin changes in vivo in a controlled setting.

## 2 Materials and Methods

### 2.1 Study Design

This pilot study investigated the feasibility of the SCAI‐app for detecting simulated skin changes. The study was carried out in the Danish Research Center for Skin Cancer at Department of Dermatology, Private Hospital Molholm, Vejle, Denmark in the 1st quartile of 2024.

Healthy adults with Fitzpatrick skin type I‐III were included on a volunteer basis. Volunteers with visible skin diseases or tattoos on back or lower legs and/or known intolerance to adhesive tape were excluded. The study was conducted in accordance with the Helsinki Declaration and adhering to ISO 14155:2020 standards for medical devices. No further approvals were required due to the inclusion of healthy volunteers and non‐invasive intervention. Informed consent for participation and image publication was obtained from all volunteers.

### 2.2 Study Materials

Simulated skin changes (test spots) with adhesive tape were manually applied to the skin on back and lower legs and images were captured with the SCAI‐app (SkinChange.AI, Denmark) both before and after test spot application. The study was conducted in a controlled environmental setting with a customized light box (TOLEDO Flex LED, Global Greentech, Denmark) with a fixed light output.

#### 2.2.1 Test Spots

The simulated skin changes consisted of adhesive test spots customized for this study, made of laminated paper on medical tape (3 M Micropore, USA) and cut‐out with a 3 mm biopsy punch (PFM, Germany). Three different colored test spots were created; black (RAL: 9005), brown (NCS: S4030‐Y30R), and red (clinical image of basal cell carcinoma). A total of eight spots were placed on each volunteer, comprising two black spots, one brown spot, and one red spot on the back and legs, respectively. See Figure 1 for test spot examples and closeup on skin as well as sketch of systematic test spot placement.

**FIGURE 1:** Test spots with respective color‐code (a) example, (b) closeup, and in (c) protocol sketch of systematic placement of test spots on back and lower legs (not to scale).

#### 2.2.2 Artificial Intelligence App

The SCAI‐app system (SkinChange.AI version 2.2.2 for iOS version 13.0 and above) consists of (a) a smartphone app interface for standardized image collection, and a backend algorithm comprising (b) AI‐assisted standardized alignment and (c) AI‐assisted comparison of paired images.

The smartphone app interface provides anatomical templates of individual body parts that guide the operator in capturing standardized images. Based on the first image, individually adjusted templates are created for a second image, allowing direct pairing of images on the screen. The template and the iOS built‐in smartphone gyroscope further secure alignment of angles as well as photographic distance. The images are saved on a host server for the AI analysis.

The first AI‐assisted standardization secures exact alignment between the paired images. First, by identifying and eliminating disturbing background features. The AI used for the background identifier is based on a convolutional neural network (CNN) DeeplabV3Plus [22] architecture with a ResNet18 encoder [23]. It has been pretrained on ImageNet dataset (1M+ images) [24] and additional training was conducted for general skin detection on 6000 images and additionally 50−200 images for each body part. Second, the AI algorithm adjusts for any remaining standardization differences between the images in three steps: (i) Misalignment of the relative position and body posture is compensated through a 3D representation. (ii) Color differences are aligned by eliminating pixel errors and adjusting for regional and local color differences. (iii) Each paired image pixel is aligned, allowing pixel by pixel comparison.

The second AI‐assisted step is spot identification. The AI compares the images before and after test spot application, identifying possible changes, marking the areas of interest with red rings. The spot identification AI is based on the CNN architecture YOLOv5s object detector [25], pretrained on the COCO [26] dataset (300k+ images). The dataset for additional training has been created from 360 images with multiple spots in each image.

See Figure 2a,b for the smartphone app interface and backend AI algorithm web‐interface.

**FIGURE 2:** SCAI interface for (a) the smartphone app and (b) the backend AI algorithm.

The utilized smartphone in this study was an iPhone 14 Pro Max and all images were collected by a single operator.

### 2.3 Outcome Measures

Outcome measures refer to the SCAI‐app feasibility for detecting study‐specific simulated skin changes, which derived from paired images, before and after application of a fixed number of test spots, and the corresponding AI‐based output of the SCAI‐app.

### 2.4 Statistics

Characteristics were presented with descriptive statistics. Sensitivity and specificity for detection of test spots were displayed as percentages with 95% confidence intervals (CI). The positive predictive value (PPV) and negative predictive value (NPV) were also estimated for the overall data. Additionally, sensitivity and specificity analysis were stratified by anatomical location, back and legs. Stratification by test spot colors black, brown, and red, respectively, was feasible for true positives and false negatives, while the numbers for false positives and true negatives were not color‐specific.

## 3 Results

### 3.1 Characteristics

A total of 24 healthy volunteers were consecutively included, while a single volunteer was excluded due to a tattoo in a study area. Study volunteers comprised both women (75%) and men (25%) with a median age of 55 and a range of 19−62 years. More than half of the volunteers presented with Fitzpatrick skin type II (54%), only a single volunteer had skin type I (4%), while the remaining had skin type III (42%).

### 3.2 SCAI‐App Output

A total of 192 test spots were placed, amounting to 96 on backs and 96 on legs. A total of five test spots were excluded from the analysis; in one patient, the back images (2 black, 1 brown, and 1 red) were not saved correctly to the server, and in another patient, one test spot (1 black) was placed too laterally for the AI detection. See Figure 3 for an example of the SCAI‐app detection output.

**FIGURE 3:** SCAI‐app output example on a volunteer's back (a) before test spot application; (b) after test spot application; (c) SCAI‐app detection with red rings. In this figure, additional arrows mark true‐positives (green) and false‐positives (red), no false‐negatives in this example.

#### 3.2.1 Sensitivity, Specificity and Predictive Values

Overall, the SCAI‐app provided test spot detection with a sensitivity of 92.0% (CI: 88.1–95.9) and a specificity of 95.5% (CI: 95.0–96.0). The overall ability to identify a true positive test spot among false positive test spots (PPV) was 38.0% (CI: 31.0−44.9) while the ability to correctly identify true negatives (NPV) was 99.7% (CI: 99.0−100). The overall number of true negatives identified by SCAI‐app was substantial (*n* = 5949).

Stratification of the data by location and test spot color revealed pertinent details of the SCAI‐app output. Sensitivity was higher on the back compared to the lower legs (back: 98.9% [CI: 96.8−100], legs: 85.3% [CI: 78.1−92.4]), while it was the opposite for the specificity (back: 93.8% [CI: 93.0−94.5], legs: 98.1% [CI: 97.5−98.6]). There was a tendency towards red and black test spots being more distinguishable than the brown (sensitivity; red: 93.6% [CI: 86.6−100], black: 92.5% [CI: 87.1−97.8], brown: 89.4% [CI:80.5−98.2]). See Table 1 for overview of sensitivity and specificity analysis.

**TABLE 1:** Sensitivity and specificity analysis of the SCAI‐app output in percentages with 95% confidence intervals (CI) and absolute numbers; overall, by anatomical location and color‐code, respectively.

SCAI output	Spots	Spots by location		Spots by color‐code		
Test spots	Overall (*n* = 187)	Back (*n* = 92)	Legs (*n* = 95)	Black (*n* = 93)	Brown (*n* = 47)	Red (*n* = 47)
**Sensitivity % (95% CI)**	92.0% (88.1−95.9)	98.9% (96.8−100)	85.3% (78.1−92.4)	92.5% (87.1−97.8)	89.4% (80.5−98.2)	93.6% (86.6−100)
**Specificity % (95% CI)**	95.5% (95.0−96.0)	93.8% (93.0−94.5)	98.1% (97.5−98.6)	95.5% (95.0−96.0)	94.8% (94.2−95.4)	95.1% (94.4−95.7)
**Absolute numbers, *n***						
**True positive**	172	91	81	86	42	44
**False negative**	15	1	14	7	5	3
**False positive**	281	233	48	281^*^	281^*^	281^*^
**True negative**	5949	3495	2454	5949^*^	5949^*^	5949^*^

* Not color‐specific.

## 4 Discussion

This pilot study sought to investigate the detection skills of a novel smartphone app‐based AI system, SCAI‐app. Overall, the app provided in vivo detection of the study‐specific test spots with a sensitivity of 92.0% and specificity of 95.5%. Meanwhile, a PPV of 38.0% and a NPV of 99.7% indicated that the app rarely overlooked the simulated skin changes, but a substantial part of marked possible areas of interest were not actual changes. Balancing false negatives and false positives is a general tradeoff and presents a substantial challenge in tools such as the SCAI‐app. While, a low rate of false negatives is crucial to relevant detection of skin changes, a high rate of false positives presents other considerable challenges that are important to address. Overestimation of possible skin changes may induce significant unnecessary worry in individuals operating such an AI tool. In extension, the handling and differentiating of false positives may give rise to an additional, increasing overload of the health care systems, which counteracts the application of AI‐assisting tools for skin checks.

This study provided important learning points for optimization of the SCAI‐app. Generally, detection was better on the back compared to the lower legs, which could be explained by several factors. First, images of the lower legs were captured from a longer distance than those of backs, and therefore the spots consisted of fewer pixels, making them harder to track with the fixed study settings and the current AI‐training status. Second, the background identifier AI was more precise in border definition of the back compared to the legs, which caused the system to exclude spots on legs as background features. Post‐analysis investigations showed that the AI‐system performance could be further enhanced with minor setting adjustments and additional AI training.

### 4.1 Perspectives

Detection of skin changes is challenging as well as time‐consuming and resource‐heavy [6, 7]. Individuals may struggle to identify new or growing skin lesions, especially on large or unattainable areas of skin such as the back. Additionally, skin types with multiple skin lesions or severely pigmented and sun‐damaged skin may be even more demanding in regard to skin checks [27].

Currently, tools for assisting identification of skin changes mainly exist in passive forms, comparing still‐images over time [28]. However, this leaves the identification of new or changing skin lesions entirely up to the eye of the beholder, which can be anything from a non‐trained individual to dermatology novices or dermatologists [29, 30]. Moreover, image quality is crucial for optimized AI application but remains challenging. While newer smartphone applications such as the SCAI‐app have taken steps toward improved image standardization, the image acquisition techniques of available tools have proven to vary substantially [12]. In a wider perspective, AI systems such as the SCAI‐app may potentially prove to be useful in democratizing early detection of skin lesions, especially in regions where clinical assessment is unavailable or sparse. However, AI‐tool limitations are important to consider in future implementation [12].

Compared to other AI systems within skin lesion detection [17, 20, 21, 31], the SCAI‐app was trained based on identification of non‐specific spots. Potentially the SCAI‐app could be applicable to a variety of skin lesions, as it is more broadly trained to non‐discriminatorily detect skin changes instead of specific clinical features. However, the possibility to apply the SCAI‐app in less controlled settings as well for detection of actual clinical lesions is yet to be investigated in a clinical trial.

## 5 Conclusion

Overall, the SCAI‐app presented sensitivity of 92.0% and specificity of 95.5% for in vivo detection of the simulated skin changes. The SCAI‐app showed a particular identification of true negatives (NPV 99.7%) and less precise distinction between true and false positives (PPV 38.0%), representing the challenging tradeoff between false negatives and false positives.

Based on this pilot study, the SCAI‐app may potentially prove relevant as an AI assistant for skin checks. However, the clinical feasibility remains to be investigated in a trial with clinical skin lesions.

## Ethics Statement

The study was conducted according to the guidelines of the Declaration of Helsinki and ISO 14155:2020 standards for medical devices.

## Conflicts of Interest

B.V. is a shareholder and employee at SkinChange.AI Aps.

## Informed Consent Statement

Informed consent was obtained from all subjects involved in the study.

## Data Availability

A data compilation presented in this study is available upon request from the authors. Raw data based on images on host server cannot be shared due to GDPR‐agreement (Edora A/S).
